The article "Effect of Methomyl on Growth, Antioxidant System of GIFT (Oreochromis niloticus), and Residue in the Presence of Water Spinach (Ipomoea aquatica Forsk)" was published in 2022. Journal: Int J Anal Chem.

# Effect of Methomyl on Growth, Antioxidant System of GIFT (*Oreochromis niloticus*), and Residue in the Presence of Water Spinach (*Ipomoea aquatica* Forsk)

**DOI:** 10.1155/2022/7434426

**Published:** 2022-08-12

**Authors:** Xiaojun Jing, Yao Zheng, James P. Mulbah, Jiazhang Chen, Gangchun Xu

**Affiliations:** ^1^Key Laboratory of Integrated Rice-Fish Farming Ecology, Ministry of Agriculture and Rural Affairs, Freshwater Fisheries Research Center (FFRC), Chinese Academy of Fishery Sciences (CAFS), Beijing, China; ^2^Wuxi Fishery College, Nanjing Agricultural University, Wuxi Jiangsu 214081, China

## Abstract

This study was conducted to investigate the effect of methomyl (MET) on the growth and antioxidant system of GIFT (5.28 ± 0.12, *n* = 180) in the presence of water spinach (*Ipomoea aquatica*) aas a floating bed. Four treatment groups have been established, named control (0), 2, 20, and 200 *μ*g/L MET. Results showed that at moderate temperatures such as 25°C to 30°C, tilapia's feed consumption increased and body weight improved. SOD, CAT, and GSH in the liver of GIFT indicated the significant increase under MET exposure. MET reduced the growth rate of GIFT, and water spinach reduced part of the water quality indexes in the MET (<200 *μ*g/L) groups. Water spinach altered GIFT's hepatic oxidation system to some extent and effectively absorbed MET in water and transferred it to itself, and the degradation time was lower than the dietary standard time which termed as 15–20 days. Growing water spinach in farmed waters partially decomposes MET and prevents it from causing damage to GIFT's liver.

## 1. Introduction

Methomyl (MET) is a broad-spectrum pesticide that is used to get rid of insect pests. The main routes of agricultural pesticide transport to different aquatic ecosystems are through drains from agricultural fields, spray drifts, disposal through wastes, and deliberate use in aquatic environments. MET (C_5_H_10_N_2_O_2_S) is S-methyl-1-N-[(methylcarba-moyl)-oxy]-thioacetimidate, classified as the most toxic and hazardous pesticide by the WHO and EPA, which is functionally analogous to organophosphates for inhibiting enzyme activity of acetyl cholinesterase in mammals and insects. MET is considered to be highly toxic to fish and aquatic invertebrates [1, 2]. The LC_50_ values for crucian carp ranged from 0.9 to 3.4 mg/L, and the LC_50_ values for *Daphina magna* were from 0.022 to 0.026 mg/L [3]. Previous studies were conducted on the effects of MET pesticides on several fish species such as *Channa striatus* [4] and tilapia (*Oreochromis niloticus* [5, 6]. The results showed that there were significant changes in antioxidant activities and contents in serum (increases in GST, GR, GPx, and GSSG accompanied by a decrease in GSH were observed following MET exposure to 2, 20, or 200 *μ*g/L). As well as in the liver, the results showed significant increases in the activities of GST, GR, and GPx and levels of GSSG accompanied by a decrease in GSH levels.

The article "Effect of Methomyl on Growth, Antioxidant System of GIFT (Oreochromis niloticus), and Residue in the Presence of Water Spinach (Ipomoea aquatica Forsk)" was published in 2022. Journal: Int J Anal Chem.

Oxidative stress is an imbalance between the production of reactive oxygen species (ROS) and the cell's ability to reduce ROS, and MET can cause an increase in ROS production in the cells of the exposed organisms [5]. On the basis of line of defense, antioxidants can be categorized as first-line defense antioxidants, SOD, CAT ,and GPx which dismutate superoxide radical, breakdown hydrogen peroxides, and hydroperoxides into harmless molecules (H_2_O_2_/alcohol and O_2_). GSH reduces H_2_O_2_ and lipid hydroperoxides with the GPx enzymes, which is an important part of the integrated antioxidant system and maintains other nonprotein antioxidants in their reduced and biologically significant state.

Water spinach (*Ipomoea aquatica*) is one of the effective aquatic plants that is used for heavy metal removal from water. We constructed the determination method for MET in plants [6], and this plant shows significant nutrient removal [7, 8], antioxidant activities [9], and immune effects [10]. However, limited information on the capability of the genus *Ipomoea* as a part of the biofilter is documented. Thus, reactive oxygen species (ROS) induced in aquatic ecosystems through pollutants can be evaluated via antioxidant enzyme activity measurement and could be excellent biomarkers [11]. Genetically improved farmed tilapia (GIFT) is suitable for culture in warm waters, but is sensitive to aquatic environmental factors [5, 6]. The present study aims to investigate nutrient removal and water quality of tilapia wastewater using water spinach as a floating bed; to know the effect of a chronic sublethal dose of MET on growth performance (BWG, SGR, and FCR) of GIFT; and to investigate the effect of a chronic sublethal dose of MET on antioxidant enzyme activities (SOD, CAT, GPx) and GSH content in the liver of GIFT. The present study hypothesized that growing with water spinach may have a positive effect on the prevention of GIFT's liver toxic damage.

## 2. Materials and Methods

### 2.1. Experimental Design and Sampling

MET was obtained from Shanghai Focus Biological Technology Co., Ltd, China (98% purity, with miscible oil <2%) and dissolved in pure water to form stock solutions, and then the experimental concentration in aquariums was diluted immediately before use. The study applied a static system with a floating bed. A total of 12 glass aquaria (40 cm × 40 cm × 60 cm, and 100 L) were used. Erstwhile to use, mint height of 10 cm was planted in several floating pots and placed in a tank. Mint was stored in a 1000 cm^3^ tank in 300 L of water and acclimated to wetland conditions for four weeks. There was no artificial nutrient addition for mint during the acclimatization and the experiment. Juveniles of GIFT (*n* = 500) were obtained from the fish farm in the Yixing research center of FFRC-CAFS, China. Before the experiments, the fish were acclimated under laboratory conditions. After four weeks, the fish were transferred to the aquarium. The commercial feed (the moisture, crude protein, crude lipid, and energy were 4.78%, 46.42%, 8.19%, and 14.31 Mg/kg, respectively) was purchased from Jiangsu Zhe Ya Food Co. Ltd., China. Fish were fed twice daily with commercial feed (extruded pellets), and the feeding rate was 5% of total body weight. This ration size was built on preliminary observations to drive the fish to feed on the roots, stems, and leaves of mint, also to prevent water quality deterioration, as well as for cost-saving. The experiments started when no mortality was observed in the acclimated population. Water spinach was placed at the surface of all twelve tanks at 800 g using plastic floaters.

The article "Effect of Methomyl on Growth, Antioxidant System of GIFT (Oreochromis niloticus), and Residue in the Presence of Water Spinach (Ipomoea aquatica Forsk)" was published in 2022. Journal: Int J Anal Chem.

Absolute weight gain (BWG) = final body weight (*W*_*t*_)–initial body weight (W_0_). Relative body weight growth rate (BWG, %) = (*W*_*t*_ − *W*_0_)/*W*_0_ × 100. Specific growth rate (SGR, 100%) = (ln*W*_*t*_–ln*W*_0_)/(*t*_2_-*t*_1_) × 100. Feed conversion rate (FCR) = dry feed fed/body mass gain where *t*_1_ represents the initial time of the test and *t*_2_ represents the end time of the test. The SGR assumes an exponential growth of fish over the whole life cycle, which is incorrect. Fish growth rate is weight dependent and, therefore, SGR will vary over different life stages of fish (i.e., lower with increasing weight). Therefore, SGR may not be a suitable parameter in comparing the growth of fish between different studies. Feed conversion is the total of nutrients accumulated into tissue for weight gain. It covers all of the nutrients. FCR depends on the composition of the diet, quantity of feed, feeding frequency, age, and species of fish.

A set of juveniles were randomly distributed into 1500 L plastic tanks containing 750 L of water with different MET sublethal concentrations as follows: 0, 2, 20, and 200 *μ*g/L (12 tanks for 4 groups in triplicate). Fifteen fish were introduced in each concentration in an open-static system with the total experimental fish of 180 (*n* = 15 per tank for different groups in triplicate). 800 g of water spinach was added to all the experimental tanks, including the control with the weight of water spinach coming up to 9600 g, and the water did not change until the end of the experiment. The entire experiment lasted for ninety days, including an acclimatization period, but the total exposure was sixty days. The first water samples were collected after 2 (named as w2), 4 (named as w4), 6 (named as w6), and 8 (named as w8) weeks of exposure to the MET concentrated water, while the fish liver samples were collected at w2, w4, and w6. All the liver samples were collected using the same format—fish caught and the weight and length recorded— they were decapitated and the liver was extracted and kept in the refrigerator at −85°C pending analysis.

The article "Effect of Methomyl on Growth, Antioxidant System of GIFT (Oreochromis niloticus), and Residue in the Presence of Water Spinach (Ipomoea aquatica Forsk)" was published in 2022. Journal: Int J Anal Chem.

### 2.2. Water Quality

Monitoring and data collection started one week after the plant and fish were acclimatized to the system. Water quality was measured daily for two weeks in aquariums. To test the mint as part biofilter, triplicate water samples from each of the treatment sets were transferred to a 500 mL polyethylene bottle to test physicochemical parameters of ammonia-nitrogen (NH_4_^+^-N), nitrite-nitrogen (NO_2_^−^-N), nitrate-nitrogen (NO_3_^−^-N), and total nitrogen (TN). All samples were filtered with a Whatman filter paper of a pore size of 0.45 *μ*m before laboratory analysis.

### 2.3. Antioxidant Enzymes Activities Determination

Taking the samples of the fish started after three weeks of exposure to the MET contaminated water. Fish were made to fast a day before sampling. Three fish each was taken from the tanks and slaughtered. The liver was extracted, weighed, and kept in a refrigerator at −85°C until analysis. Sodium chloride (NaCl) 0.9 g was dissolved in 100 ml and was used for the extraction of the supernatants. The tissues were homogenized using a portable homogenizer. 25 ml of saline solution was added to the homogenized tissue and centrifuged at 250 nm for 10 min. The supernatants were collected into a tube and kept at 4°C. This supernatant was used to carry out the assay of CAT, SOD, GSH, and protein content. The supernatants were prepared using test assay and taken to the spectrophotometer for results [12]. A spectrophotometer was used to measure the absorbance at different wavelengths (412 nm, 405 nm, 550 nm, etc.,), and a thermostatic water bath was capable of controlling temperature at 37°C.

### 2.4. MET Residue

The plant samples (root, stem, and leaf) were collected at two-week intervals and dried in an electrical oven at a temperature of 105°C. It was powdered using an electric grinder. The plant samples (1.5 g) were put into a 50 ml centrifuge tube, mixed with 10 mL acetonitrile and homogenized at 2500 rpm for 5 minutes, and centrifuged at 3500 rpm for 5 minutes (this was done twice), and the supernatant was transferred into a 50 mL tube and taken to the solid face extraction for further extraction. Here, 10 mL of acetonitrile-toluene (3 : 1 v/v) was used to activate the cartridge and the supernatant was filtered through the cartridge. 20 mL of acetonitrile-toluene (3 : 1 v/v) was measured, and 2 mL of the solution was used 3 times to wash the tube and added to the cartridge. The cartridge was then eluted with 19 mL of acetonitrile-toluene (3 : 1 v/v). The eluent was then collected and evaporated to dry at 40°C using the rotary evaporator. The dried residue was dissolved in 1 ml of acetonitrile and filtered with a 0.45 *μ*m organic membrane filter using a syringe, and the sample was taken to HPLC for analysis.

The article "Effect of Methomyl on Growth, Antioxidant System of GIFT (Oreochromis niloticus), and Residue in the Presence of Water Spinach (Ipomoea aquatica Forsk)" was published in 2022. Journal: Int J Anal Chem.

### 2.5. Data Analysis

The data collected was analyzed by one-way ANOVA using the Statistical Package for Social Sciences (SPSS 26.0) to determine the level of CAT, SOD, and GSH in GIFT. GSH was expressed as nmol GSH/mg protein. The data are presented as mean ± SE values. The numbers of animals per group were stated in the table or figure legends. The statistical analysis of the data was performed using one-way analysis of variance (ANOVA). The significance of the results was ascertained at *P* < 0.05 with a lowercase letter.

## 3. Results

### 3.1. Water Quality

There was no significant difference (*P* > 0.05) in FCR and SGR at the treatment group 2 and 20 *μ*g/L exposed to MET sublethal concentrated water as compared to control group, but there was a significant increase (FCR) and decrease (SGR, *P* < 0.05 between treatment 200 *μ*g/L fish exposed to MET sublethal concentrated water and the control treatment, and there were some significant difference (*P* < 0.05) within groups (Table 1).

TN (except w8) and NO_3_^−^-N in the control group were significantly higher than those in other groups (Figure 1(a)), while TN in the 200 *μ*g/L treatment group showed a significant increase when compared to the controls at w8. TN (at w6 and w8) and NH_4_^+^-N (at w2, w4 and w6, Figure 1(b)) in the 200 *μ*g/L treatment group showed a significant increase when compared to those in the 2 *μ*g/L treatment group, while NH_4_^+^-N at w8 showed the converse tendency. NH_4_^+^-N (at w2 and w6) in the 2 *μ*g/L treatment group showed a significant decrease when compared to those in the control group, while NH_4_^+^-N at w4 showed the converse tendency. At w2, NO_3_^−^-N in the control treatment group showed a significant decrease (*P* < 0.05) as compared to 200, 20, and 2 *μ*g/L MET groups. At w2, NO_2_^−^-N in the 200 *μ*g/L treatment group showed a significant increase (*P* < 0.05) as compared to 20 and 2 *μ*g/L and the control groups. The NO_3_^−^-N concentrations at w4, w6, and w8 showed that there was no significant difference (*P* > 0.05) (Figure 1(c)). NO_2_^−^-N in the 2 *μ*g/L treatment group and the control groups showed a significant decrease (*P* < 0.05) as compared to the 20 and 200 *μ*g/L treatment groups at w2 (except for 20 *μ*g/L, Figure 1(d)) and w6.

The article "Effect of Methomyl on Growth, Antioxidant System of GIFT (Oreochromis niloticus), and Residue in the Presence of Water Spinach (Ipomoea aquatica Forsk)" was published in 2022. Journal: Int J Anal Chem.

### 3.2. Oxidation Enzyme Activities

The effect of SOD in the liver of GIFT indicates a significant increase (*P* < 0.05) in the 2 *μ*g/L treatment group compared to the other treatment group at w4 (except for 20 *μ*g/L, Figure 2(a)) and w6. SOD in 2, 20, and 200 *μ*g/L-w2 showed a significant decrease (*P* < 0.05) compared to the control group.

Glutathione was a good antioxidant enzyme and was vigorous against oxidation in living things. The presence of CAT in the liver of GIFT has shown a significant difference (*P* < 0.05) at w4 and w6 as compared to those at w2 (Figure 2(b)). In the 2 *μ*g/L treatment group, w4 was significantly higher (*P* < 0.05) compared to the other treatments. At w6, CAT in the 200 *μ*g/L group was significantly lower (*P* < 0.05) as compared to the other treatments, whereas CAT in the 2 and 20 *μ*g/L groups significantly decreased and increased (*P* < 0.05) compared to the control and 200 *μ*g/L treatment groups, respectively.

In the above GSH graph (Figure 2(c)), there were significant differences (*P* < 0.05) at w2, w4, and w6. GSH in the 200 *μ*g/L treatment group at w2 significantly decreased (*P* < 0.05) compared to other groups at w2, and there was no significant difference between lower groups at w2. A significant increase of GSH occurred in the 20 *μ*g/L group at w4/6 compared to 0, 2, and 200 *μ*g/L groups, while GSH in the 2 *μ*g/L group at w4/6 was significantly higher than those in the control (including 200 *μ*g/L group at w6) groups.

### 3.3. MET Residue

In this section of study, water spinach was exposed to MET solution at various concentrations for 60 d. The samples of the plants were collected from the roots and evaluated to establish the significance of the pesticide residue in the plant.

The MET residue in roots of the control groups in all the weeks significantly increased than those in the other groups (Figure 3(a), *P* < 0.05). MET residue in the 2/20/200 *μ*g/L treatment groups at w2 showed a significant increase than the controls, while w1 revealed no significant difference among each group. MET residue in the 20/200 *μ*g/L treatment groups at w4 (with no significant difference in 20/200 *μ*g/L groups) and w6 (in a dose-dependent manner) significantly decreased and increased (*P* < 0.05) as compared to the 2 *μ*g/L groups, respectively. After w6 MET exposure, the MET residue had significantly increased with the increased concentrations.

The article "Effect of Methomyl on Growth, Antioxidant System of GIFT (Oreochromis niloticus), and Residue in the Presence of Water Spinach (Ipomoea aquatica Forsk)" was published in 2022. Journal: Int J Anal Chem.

The residual ability of MET in the stem of the water spinach at w2 (*P* > 0.05 among three MET groups), w4 (*P* > 0.05 among three MET groups), and w6 in the treatment groups showed significant increase (Figure 3(b), *P* < 0.05) as compared to those in the control group, while MET residue in the 20 *μ*g/L treatment group showed no significant difference as compared to those in the 2 *μ*g/L treatment group. The MET residue in the 200 *μ*g/L groups significantly increased compared to those in the 2/20 *μ*g/L groups. The similar tendency is also seen in the leaves at w2/4, and only MET residue at w6 showed a significant increase (Figure 3(c), *P* < 0.05) in leaves with the dose-dependent manner.

## 4. Discussion

Water quality may affect fish's health when under toxicant exposure, and the present study showed the detected parameters in the 200 *μ*g/L MET group were without significant differences at w4/6/8 except for NH_4_^+^-N (w4/8) and NO_2_^−^-N (w6). The antioxidant enzymes at w4/6 also showed the same tendency except for CAT (w6) and GSH (w4) when compared to the short-term exposure duration. The FCR and SGR showed a significant increase and decrease in the 200 *μ*g/L MET when compared to the controls. This experiment indicates that the highest concentration of MET sublethal dose (200 *μ*g/L) in water did not badly affect the fish, but there was a slower pace of growth in the fish with the highest concentration of the pesticide. From observation during feeding, all feed was consumed by the fish, and because of this, parameters like ammonia, nitrite, and nitrate, were at very low concentrations in the fish tanks. Another contributing factor would be natural environmental factors such as the tanks exposure to nature. It was also observed that fish eat the roots of the water spinach that had been placed in the tanks, which has turned out to be one of the health benefits. The MET residue in the root, leaf, and stem showed a significant increase in the MET exposure groups when compared to the controls, and especially revealed a dose-dependent manner at w6. The plants eaten by the fish helped to revamp their immune systems, which induced a higher production and more healthy status [13–15]. Recent papers demonstrated that taurine [16] and parsley (*Petroselinum crispum*) seed meal alleviated MET-adverse impacts on tilapia growth [17]. Our previous studies showed that dietary resveratrol supplementation alleviated hepatic impairment through inflammatory response prevention [12] and intestinal health enhancement [18]. It was also important to know that the higher the concentration of MET, the lower the FCR and the slower the growth rate in future studies.

The article "Effect of Methomyl on Growth, Antioxidant System of GIFT (Oreochromis niloticus), and Residue in the Presence of Water Spinach (Ipomoea aquatica Forsk)" was published in 2022. Journal: Int J Anal Chem.

Pesticides have been identified to cause overproduction of ROS, which if not thoroughly neutralized by antioxidant mechanisms, may lead to oxidative stress and potential tissue damage [5]. The increased lipid peroxidation demonstrated in MET-treated mice [19] is in line with the previous study in which carbamates and their degradation products were reported to act on membranes, oxidizing their lipid components and. Some authors stated that there was a lack of effect in CAT levels in the gills of fish exposed to carbamates [20], appearing only after exposure to high concentrations. However, reduced CAT levels were found in *C. punctatus* exposed to pyrethrins [21]. Gills are the first point of contact with xenobiotics, yet they do not always have an effect on this tissue. They pass directly through this barrier and act on other tissues like the liver. Meanwhile, CAT levels were reported to be higher in the liver because they are responsible for breaking down toxins present in the blood and processing metabolic products for degradation [22]. Different pesticides induced hepatic CAT activity during the first 48 h of exposure, and likewise, it was observed that rainbow trout exposed to 25 *μ*g/L of carbamate carbosulfan for 60 days greatly increased the liver CAT activity when compared to controls [23].

Equally so, oxidative stress levels in fish from waters contaminated by different concentrations of pesticides were totally different, and in some cases a clearly inhibitory effect was experienced. The study observed a decrease in CAT activity in the liver of silver catfish exposed to the herbicide clomazone. There were similar effects found in the liver of the freshwater fish *Channa punctatus* tested after 24 h of treatment with endosulfan [24]. The study also realized a significant decline in CAT activity in zebrafish subjected to atrazine. Curiously, this same xenobiotic was assayed, who noticed an increase in the liver CAT activity after the exposure of *C. punctatus*. The first line of defense against oxidative stress comprises antioxidant enzymes (e.g., CAT), and a decrease in their activity alters the redox status of the cells. It is therefore possible that an increase in the activity of the enzymes contributes to the elimination of ROS induced by cells exposed to pesticides. GSH is also widely used as an environmental biomarker [25]. In some studies, hepatic GSH activity lessened after a few days of exposure to different kinds of pesticides [26]. In accordance with this, the liver of fish fed with a standard diet and exposed to the herbicide quinclorac showed a marked inhibition of GSH activity [27]. Nevertheless, other studies have also observed an opposite effect, for example, low levels of exposure of *Clarias gariepinus* to fenthion formulations resulted in the induction of the liver GSH activity [28]. The present study showed the increased SOD and the compensating effect of CAT (decrease) under MET exposure, while the increased GSH (*P* < 0.05) occurred in 2/20 *μ*g/L MET groups, accompanied by the subsequent decrease in the form of homeostasis balance. The present study suggested that growing with water spinach may have a positive effect on the prevention of GIFT's liver toxic damage. Whether the eating of water spinach by tilapia may be attributed to the positive effect should be determined.

The article "Effect of Methomyl on Growth, Antioxidant System of GIFT (Oreochromis niloticus), and Residue in the Presence of Water Spinach (Ipomoea aquatica Forsk)" was published in 2022. Journal: Int J Anal Chem.

Results showed that the roots and the leaves were more affected by the pesticide as compared to the stem. At w4 and w6 of the experiment, MET residual potential in the root was of significant difference as compared to those at w2. Results from the stem indicate that only w6 showed a significant difference (*P* < 0.05). There was no significant difference at w2 and w4. The leaf, which was one of the most important parts of this economical plant does not have much significant difference, and only MET residues at w6 also showed a significant difference (*P* < 0.05). MET was revealed in the liver and muscle of fish [29], and the current study indicated that *Ipomoea aquatic*, when exposed to MET-concentrated water, had some MET absorption effects on the plant.

Supervised residue data from trials in several other countries showed that MET  residues were detected on most above-ground crops at the time of harvest [6]. Higher residues occurred on leafy vegetables, for example, lettuce, spinach, celery, and cabbage, with generally low levels on root crops, cucurbits, and grain crops. High residues were detected in alfalfa, pea, bean, and peanut foliage and straw of wheat, oats, and barley [30, 31]. The residue level diminished with time after application. The amount of insecticide was applied, time interval between last application and harvest, surface area, weight, and surface structure of the crop were factors that affected the level of the residue [32]. The amounts of residue resulting from the use of the powder and liquid formulations were nearly identical when an equal amount of active ingredient is applied. The degradation of MET was lower than the dietary standard through 15–20 days in the present study, which suggested that fish farmers should sell water spinach during the harvest to obtain the added value.

## 5. Conclusions

MET reduced the growth rate of GIFT, and water spinach decreased part of the water quality indexes. SOD, CAT, and GSH were significantly decreased in 200 *μ*g/L groups, while those activities were increased in 2 *μ*g/L groups, especially GSH after long-term MET exposure duration. Water spinach is a good source of nutrients that accumulate toxic residue, especially in the root and the leafy parts. The degradation time of MET was lower than the dietary standard time, which was termed 15–20 days.

The article "Effect of Methomyl on Growth, Antioxidant System of GIFT (Oreochromis niloticus), and Residue in the Presence of Water Spinach (Ipomoea aquatica Forsk)" was published in 2022. Journal: Int J Anal Chem.

## Figures and Tables

**Figure 1:** The water quality indexes in experimental tanks during different weeks. Total nitrogen (TN) (a), ammonia (NH_4_^+^-N) (b), nitrate (NO_3_^−^-N) (c), and nitrite (NO_2_^−^-N) (d) were revealed with the unit of mg/L. The treatment for 0, 2, 20, and 200 *μ*g/L MET in triplicate (n = 12 total tanks for 4 groups and n = 15 individuals per tank in triplicate).

**Figure 2:** Combined view of SOD, CAT, and GSH concentrations in the liver of GIFT exposed to MET contaminated water at w2, w4, and w6. Different subscripts in each group indicate significant difference. The treatment for 0, 2, 20, and 200 *μ*g/L MET in triplicate (n = 12 total tanks for 4 groups and n = 15 individuals per tank in triplicate).

**Figure 3:** Combined view of MET  residue in the root, stem, and leaves of the water spinach at w2, w4, and w6. Different subscripts in each group indicate significant difference. The treatment for 0, 2, 20, and 200 *μ*g/L MET in triplicate (*n* = 12 total tanks for 4 groups and *n* = 15 individuals per tank in triplicate).

**Table 1:** The effects of biological parameters under different concentrations of MET exposure.

Group	Control	2 *μ*g/L	20 *μ*g/L	200 *μ*g/L
*W*_0_(*g*)	5.32 ± 0.06	5.31 ± 0.07	5.09 ± 0.09	5.25 ± 0.10
*W*_*t*_(*g*)	33.52 ± 0.35	31.79 ± 1.37	30.11 ± 1.24	28.83 ± 1.08
WG	529.39 ± 9.25	498.67 ± 29.77	491.24 ± 22.37	449.48 ± 28.38
FCR (%)	1.06 ± 0.01^b^	1.13 ± 0.06^ab^	1.20 ± 0.05^ab^	1.27 ± 0.06^a^
SGR (%/day)	3.06 ± 0.02^a^	2.97 ± 0.08^ab^	2.95 ± 0.06^ab^	2.83 ± 0.08^b^

Note: The initial weight, final body weight, weight gain, feed conversion ratio, and specific growth rate were named as W_0_, W_t_, WG, FCR, and SGR, respectively. The significance of the results was ascertained at *P* < 0.05 with a different lowercase letter.

## Data Availability

The data used to support the findings of this study are included within the article.
